# Recent Applications of Electrospun Nanofibrous Scaffold in Tissue Engineering

**DOI:** 10.1155/2022/1953861

**Published:** 2022-02-09

**Authors:** Hamza Abu Owida, Jamal I. Al-Nabulsi, Feras Alnaimat, Muhammad Al-Ayyad, Nidal M. Turab, Ashraf Al Sharah, Murad Shakur

**Affiliations:** ^1^Medical Engineering Department, Faculty of Engineering, Al-Ahliyya Amman University, Amman 19328, Jordan; ^2^Department of Networks and Information Security, Faculty of Information Technology, Al-Ahliyya Amman University, Amman 19328, Jordan; ^3^Computer Engineering, Faculty of Engineering, Al-Ahliyya Amman University, Amman 19328, Jordan

## Abstract

Tissue engineering is a relatively new area of research that combines medical, biological, and engineering fundamentals to create tissue-engineered constructs that regenerate, preserve, or slightly increase the functions of tissues. To create mature tissue, the extracellular matrix should be imitated by engineered structures, allow for oxygen and nutrient transmission, and release toxins during tissue repair. Numerous recent studies have been devoted to developing three-dimensional nanostructures for tissue engineering. One of the most effective of these methods is electrospinning. Numerous nanofibrous scaffolds have been constructed over the last few decades for tissue repair and restoration. The current review gives an overview of attempts to construct nanofibrous meshes as tissue-engineered scaffolds for various tissues such as bone, cartilage, cardiovascular, and skin tissues. Also, the current article addresses the recent improvements and difficulties in tissue regeneration using electrospinning.

## 1. Introduction

The biomedical industry has contributed on a large scale with technologies in treatment that has led to healthier lives in patients. However, recently, the biomedical sector has its focus diverted to a technology that is rather fascinating and very promising for the future of treatment [1–3]. Tissue engineering has caught the attention of many domains that have collaborated to find new solutions to produce cells and tissues naturally in the laboratory [4].

Tissue engineering is an ever-evolving technology like any other promising method for treatment, in engineering terms; it is referred to as tissue engineering [4]. However, it is also referred to as regenerative medicine. This type of treatment in the medical field is the way to the future of medicine and the biomedical field for reasons such as the disuse of medication and drugs and the growth of cells in the lab that are mainly from the body to the body of the subject [4–6]. Therefore, it is highly unlikely to be rejected by the body's immune system. Nevertheless, it is unfortunate that at the moment, the process of tissue engineering or regenerative medicine is costly and time-consuming [5, 7]. However, the collaboration of many medical and biomedical fields is working on enhancing the tissue engineering process and making it more efficient to be used in treatment [8]. There are substantial challenges when it comes to tissue engineering; one of which has a rather high significance which is constructing an artificial environment to grow the desired tissue [7]. The collaboration mentioned earlier focuses on enhancing the scaffold that the tissue would grow in; the main goal in this research is to find the most efficient method for the biocompatible scaffold to allow the tissue to grow completely without burdens and complications [4]. Hence, the main function of the scaffold is to host that desired tissue and allow for natural growth until it is ready to be introduced to a subject or patient [9]. The contribution has many technologies involved, with nanotechnology having played a key role in improving the scaffold; the more efficient the scaffolds are the better the results of the tissue [10]. There are many types of scaffolds and there are many ways to construct them, which are then used to obtain tissue growth. However, our focus will be on the electrospinning method that has proved to be the most reliable and sustainable considering its properties [10, 11]. Nevertheless, the main goal is to ensure cell growth and survival. Tissue engineering brings on this challenge, and the initial steps are to construct a biocompatible scaffold [5, 10]. This review presents an overview of efforts to create nanofibrous meshes as tissue engineered scaffolds for a variety of tissues including bone, cartilage, cardiovascular, and skin tissues. In addition, the current article discusses the benefits and drawbacks of using electrospinning for tissue regeneration.

## 2. Setup and Procedure of a Conventional Electrospinning System

The main reason for the focus on the electric spinning method is to use its reliability in the production of nanofibrous biomaterials. The technology is sophisticated, yet it is easy to understand how it works, especially the process in the biomaterial production. Nevertheless, it is not a new technology; it was used around the century ago; however, it has successfully caught the attention of researchers and scientists recently and it is being adopted to produce the scaffolds that will host this successful growth of the desired tissue [12]. To simply illustrate what happens in the electrospinning method, the liquid is highly charged. Together with a pin with an opposite charge, it then causes a discharge of a thin layer of the solution; as it is flying off the pin, it dries out to a solid state creating a mesh of the biomaterial that is very thin as shown in Figure 1 [12]. These size and dimension serve very well in tissue engineering; with a high surface area, it allows the tissue to grow naturally and efficiently [12, 13]. The electrospinning process allows for a constant scaffold production with the same consistency of the material with a higher surface area; the scale needed for the nanofibrous production in this method remains uniform throughout its production [13, 14]. There are a lot of methods and technologies for creating scaffolds; some of which have proved to be very reliable. One example is 3D printing. It can create the scaffolds with a low uncertainty in the dimensions needed; however, it is very expensive and the rate of production is rather lower. Another example is selective laser sintering that is approximately as accurate as 3D printing; nevertheless, it has the same disadvantages as 3D printing [15–17]. To sum up, electrospinning is an easy-to-use, fast, and efficient method to produce biomaterial scaffolds by applying a high-voltage electric field difference to the solution, which is then easily collected to be used in the growth of tissues in the laboratory. Definitely, electrospinning is an ideal method for tissue engineering [11, 12].

## 3. Parameters' Influence on Electrospinning Process

A number of factors influence the diameter and morphology of electrospun nanofibers, including polymeric solution properties, processing parameters, and ambient conditions [18].

The morphology and diameter of electrospun nanofibers are strongly influenced by the polymeric solution properties (such as concentration, viscosity, and the solution surface tension) [19]. The electrospinning process is heavily reliant on the concentration of the solution; hence, only a minimal amount of solution is required to run the electrospinning device [20]. Nanofibrous biomaterials can only be created by electrospinning if the solution concentration is just right during the procedure. Low-concentration solutions can result in the formation of unwanted droplets as a result of surface tension effects [21]. In addition, the high viscosity of the solution fiber structure would provide a challenge at large concentration of the material. Increases in polymer concentration may also result in fiber diameter production [22]. The size and shape of the fibers can also be highly impacted by the solution's viscosity. Electrospinning requires a viscosity that is just right so that homogeneous and fine fibers cannot be molded in low-viscosity solutions, while a continuous jet renders generating fibers impossible in high-viscosity solutions [22, 23].

Electrostatic repulsion of surface charges and the charge density force exerted by the external field are two of the principal electrostatic forces acting on a polymeric droplet at a high voltage. Such forces cause the droplet's morphology to change from spherical to conical (Taylor cone) when the voltage hits a crucial level [24]. Electrospinning and fiber fabrication can be affected by a solvent's proper surface tension, which is a function of its nature [25]. An unsteady jet and dispersion of droplets in a solution with a high surface tension can inhibit the development of fibers [26]. At lower electric fields, electrospinning can be facilitated by decreased surface tension [27].

Electrospinning process parameters (such as applied voltage, the distance between the needle and the collector, and the flow rate of the polymer solution) are another significant category in the electrospinning fabrication process [28]. In order to produce fibrous scaffolds, the process of electrospinning must overcome a threshold voltage that creates significant charge differences in the solution [29]. The development of droplets and beads in the fibers can be varied by adjusting the voltage and, consequently, the charge quantity [30].

Polymer solution flow rate is an additional consideration in this context. The time required for solvent evaporation increases when the input rate is reduced [31]. The use of a reduced flow rate in electrospinning ensures that solvents from nanofibrous scaffolds are completely evaporated [32]. Spherical fiber diameter and shape are influenced by a variety of factors, including length between needle and collector [33]. There is a difference between fibers with big average diameter and fibers with small average diameter when the distance between the collector and the fibers is large [34]. To avoid bead formation, it is important to select an optimum concentration of solution, the voltage applied, and the distance between the tip and the collector.

Electrospun sheet fabrication requires consideration of environmental conditions such as humidity and temperature, especially when dealing with difficulty in creating homogeneous fibrous sheets. The fabrication process is slowed and charging jetting is prolonged when the humidity is considerable [35]. Humidity also has a negative correlation with the solidification time. Solvents can be eliminated completely by evaporation if the humidity is low enough, although the production of fibrils can be impaired in humid settings [36]. Nanofibrous scaffolds' morphology is also influenced by temperature. Beads, which are formed at low temperatures, and condensed and flat fibers, which are formed at high temperatures, are detected [37]. Temperature increases the viscosity of the polymer solution, resulting in fibers with a smaller diameter [37]. The effects of electrospinning parameters on the resulting fiber shape are summarized in Table 1.

## 4. Developed Electrospinning Methods

The traditional electrospinning could fabricate nanofibrous structures which are determined by the shape of the collector, and the collector's angular velocity can be used to govern fiber alignment from random to precise [38].

Coaxial electrospinning, like conventional electrospinning, uses a coaxial sprayer, in which there are two different-sized spinners, one of which wraps around the other [39]. The core polymeric spray is shuttled by an inner diameter smaller than the larger one, while the shell solution is transported by the nozzle with the bigger interior diameter. The case polymeric spray and the core polymeric spray, to be pumped at the same time from two distinct storage tanks, the core-shell nanofiber and the spinner is generated who used the identical process equally conventional electrospinning via the voltage differential [40, 41]. Since only the shell polymeric spray should be electrospun in coaxial electrospinning, the electrospun biopolymers can implement nonelectrospun drugs and growth factors into their core solution [42].

Emulsification electrospinning, like coaxial electrospinning, produces core-shell structure nanofibers or doing so with polymer emulsification. This method is beneficial whereas a monospinner could indeed roll the emulsification to produce a nanofiber with several cores, without the need for an additional spinner [43]. These drops can either be resultant in nanostructure mesh to form a shape or sustain in the drops to form a multicore architecture throughout this operation. Emulsification electrospinning might be applied to fabricate nonelectrospun drugs, growth factors in polymeric solution [44].

Dynamic water flow electrospinning is a type of electrospinning in which water vortex twists nanofibers, which are then gathered on a rotary collector after being acquired on the surface of the water. An upper and lower water basin is used in this method. The water level basin has a slit in the base through that gravity turbulence could be formed on the surface of the water, if fluids flow through them. On the water's surface, the nanostructure films are first electrospun and then drip in via vortices before even being wrapped into yarn. Using a pump, liquid and yarn are pumped from the superior watershed to the minor watershed and then back to the top watershed. Porous nanoyarn scaffold is created as the yarn streams into the minor watershed and collects on a rotary collector. Tissue engineering scaffolds made from these substances have rough surfaces, wider porosities, and higher porosities than conventional electrospun nanomeshes. This suggests that they may be better suited for 3D tissue formation [45].

A different method for preparing continuous nanoyarns involves a bispray of electrospun nanofibers. Single spinner generates nanofibrous mesh with positive charge by applying a high power, while another spinner generates charges with negative polarity nanomesh by applying a negative high power. This configuration results have the effect of wrapping positively and negatively charged fibers together, which are then gathered on a rotary nozzle to shape a spiral [46].

## 5. Electrospun Nanofibrous Scaffolds for Tissue Engineering Applications

Tissue engineering is the modern way of treatment in medicine; it has achieved tremendous results with the aim of eliminating the complications that many surgical operations encounter. In engineering terms, it is called tissue engineering, derived from the processes concerning the growth of cells and tissues in the laboratory; however, it is also referred to as regenerative medicine in medical terms [4–6]. Tissue engineering combines many domains together to come up with the ultimate compensation for earlier treatment methods [5]. In a nutshell, tissue engineering is the method of growing the desired tissue or cells and then delivering the engineered tissue to the host. There are many examples of the types of tissues that are engineered, and those will be discussed thoroughly [6]. The aim of this method is to find the most suitable scaffold that will function as the support for the tissue or cells as they grow; however, there are factors to be considered in the production of the scaffolds; they should be biocompatible and biodegradable in order to be implanted to a host; moreover, factors such as size, porosity, and mechanical strength are to be considered as well [47–49]. There are various types of polymer suggested and used to produce the scaffold, biocompatible materials such as alginate, collagen, and polycaprolactone; moreover, they also have shown to have higher rates of biodegrading, with the desired dimensions to grow the tissue successfully [50–52].

### 5.1. Electrospun Nanofibrous Scaffolds for Bone Tissue Engineering

The number and variety of tissues that can be grown using tissue engineering are endless; however, there are factors that researchers have to put into consideration in order to ensure the growth of the cells or tissues [53, 54]. Engineers and researchers designing the scaffolds have priorities such as the biocompatibility which is rather referred to as step one and then comes the factor of the scaffolds being biodegradable. The scaffold must have the feature of degrading with time after being successfully delivered to the subject [55, 56]. Since this is bone tissue engineering, factors such as durability of the scaffold to remain intact upon delivery must be considered as well; therefore, the scaffold must be able to withstand ambient pressure until the cells fuse. Nevertheless, it is important that the scaffold has a high surface area that will enable the size of the scaffold to be as minimal as required [56–58]. There are many polymers that can be chosen for the manufacturing of scaffolds depending on the location of the implantation and the type of tissue grown. Polymers have the factors mentioned to successfully grow the desired bone or tissue; biomaterials that are most commonly used in bone tissue engineering are chitosan, alginate, collagen, and other polymers such as polylactic acid and polyglycolic acid [54, 59]. In particular, when it comes to bone tissue engineering scaffold concerns, researchers and engineers keep in mind biocompatibility, biodegradability, and rigidity. The scaffolds constructed must have those features when growing either bones or cartilage, since their functions in the body are mainly support and structure; the struggle is with both the growing and implantation [60, 61]. Bone tissue engineering concerning at scaffolds provides proliferation and cell attachment, which then leads to bone formation [54]. Rajzer and colleagues came up with an astonishing method where they showed that calcium phosphate osteogenic nanoparticles can be used in enhancing the scaffolds to grow bone tissue more efficiently by injecting polyaniline using an inkjet; the scaffold can be printed to improve the tissue growth [62]. Another study used hydroxyapatite due to its properties being close to the minerals of the bone; however, its fabrication with the nanofibrous scaffold also contained bone morphogenetic protein 2 and silk fibroins and using this method and scaffold able to culture mesenchymal stem cells in constant condition for 31 days; furthermore, the stem cells differentiated towards osteogenesis [63]. Samadian et al. [64] fabricated a new electrospun nanofibrous osteoconductive carbon with hydroxyapatite particles to be used *in vivo* as the scaffold for bone tissue engineering. The osteoconductive properties of the proposed nanocomposite considerably enhanced *in vivo* bone growth in the rat's femur damaged tissue. Furthermore, histological results revealed that the nanocomposite-treated group had meaningfully more bone regeneration than the damage without treatment. The results showed that the proposed fabricated nanocomposite was a potential material for bone regeneration [64]. Preeth et al. [65] introduced a bioactive zinc composite combined with polycaprolactone/gelatin electrospun nanofiber to boost bone tissue regeneration (Figure 2). Zinc is a trace mineral that is required for normal bone formation and has been shown to enhance bone formation. The authors showed that the nanofibrous mesh with zinc was biocompatible *in vivo* with high osteogenic marker expression and can be used as a therapeutic agent to repair bone defects and enhance bone formation [65]. Meka et al. [66] showed the benefit of employing strontium-eluting composite nanofibers generated by co-electrospinning nSrCO3 particles at 10% and 20% with PCL to prepare scaffolds for bone tissue regeneration. Experimental studies confirmed that the composite scaffold containing 20% nSrCO3 stimulated the growth of human mesenchymal stem cells in *vitro*. There was a significant increase in mineral deposition in PCL/SrC20, up to fourfold, indicating increased osteogenesis. As a substitute to using labile growth factors to impart bioactivity to polymer scaffolds, integration of nSrCO3 in polymer scaffolds is a viable technique for bone tissue engineering [66]. Another research by Meka et al. [67] developed a simple sol-gel technique for fabricating electrospun nanocomposite fibers in PCL using in situ silica gelation. The experimental assessment of tubular networks generated by human umbilical cord vascular endothelial cells demonstrated that eluted silicon ions and citric acid in fibers boosted angiogenic activity, which was supported by elevated gene and protein expressions of numerous known angiogenic markers. Moreover, silicate fibers promoted osteogenesis in human mesenchymal stem cells, as evidenced by enhanced mineralization and osteogenic marker gene and protein production. As a result, in situ silicated fibers are promising multi-biofunctional orthopedic composites [67]. Rajzer et al. [68] revealed a unique multifunctional layered scaffold for nasal cartilage and subchondral bone restoration made from PLLA and gelatin, as well as two scaffold production methodologies (3D printing and electrospinning). The researchers created hybrid layered scaffolds with a top gelatin nanofibrous layer and a bottom 3D-printed porous PLLA material. In simulated bodily fluid, the mineralization ability of a scaffold was assessed. Murine fibroblasts grown on acquired biomaterials were tested for cytotoxicity, proliferation, and morphology [68].

In another study, Meka et al. [69] introduced a new modified in situ sol-gel approach to create a unique multicomponent PCL nanofibrous scaffold including bioactive ceramic particles. The scaffolds improved hMSC osteogenic differentiation and HUVEC angiogenic activity. These findings show that such polymer/ceramic nanofibrous scaffolds have multi-biofunctional properties and are thus viable options for bone tissue regeneration scaffolds [69].

Gautam et al. [70] presented a new gelatin-polycaprolactone nanohydroxyapatite nanofibrous composite mesh to enhance bone tissue regeneration. DNA quantification and cell viability assays indicated decent human osteoblast viability and noteworthy proliferation rate within the proposed nanocomposite with sufficient spread of attached cells within pentagonal osteoblast morphology over the nanocomposite. As a result of the *in vitro* investigation, the proposed electrospun nanocomposite scaffold appears to be a promising applicant in order to engineer bone tissue [70].

### 5.2. Electrospun Nanofibrous Scaffolds for Cartilage Tissue Engineering

The cartilage tissue is substantial for the bodies' comfort since they act as cushions or pressure absorbents. Regrettably, the cartilage tissue takes a very long time to heal and in some cases where an injury has been undergone [71, 72]. Since it takes a long time to recover, cartilage tissue engineering is highly recommended. Scientists and researchers have constructed using the electrospinning technique with nano- and microfibrous polymer scaffolds to help in easy delivery of the tissue to the patient, and with the aid of the scaffold, it would lead for the delivered tissue to have as close as possible natural functions [73, 74]. Although there are several types of cartilage tissue, especially when considering that it will later specify certain functions, the main focus is where the cartilage has the most pressure exerted upon and ruptures from activity; therefore, it is rather significant to consider the areas within the cartilage tissue that consist of the tangential zone, which plays a crucial role since it is the superficial area of the cartilage. Moreover, the calcified zone is the thin layer heart tissue which gives the tissue its rigidity, while the transitional zone is the connection to bone or muscle. Researchers put those into consideration in order to understand the scaffold construction to ensure a successful delivery of the tissue [75, 76]. Wise and colleagues executed cartilage regeneration by adding human mesenchymal stem cells to the nanofibrous and microfibrous polycaprolactone scaffold (Figure 3); with this technique, the growing of the cartilage tissue was successful [77]. Another research also used human mesenchymal stem cells that were joined with the transforming growth factor better into the nanofibrous polycaprolactone scaffold to achieve cartilage generation due to the *in vitro* chondrogenesis being stimulated [78]. Sharifi et al. [79] fabricated an electrospun polycaprolactone combined with gelatin/chondroitin sulfate nanofibrous scaffold for cartilage tissue regeneration by chondrogenic differentiation of human bone mesenchymal stem cells without using differential medium. Cell viability assay results demonstrated a significant cellular adhesion and viability of human bone mesenchymal stem cells on fabricated nanofibrous scaffold, and the chondrogenic markers collagen type II and chondrogenic proteoglycan were expressively improved. All aided the differentiation of seeded human bone mesenchymal stem cells to chondrocytes without the use of any external chondrogenic differential factor. The fabricated nanofibrous scaffold shows better chondrogenesis differentiation outcomes and can be introduced as a viable option for cartilage tissue engineering applications [79]. Irani et al. [79] designed a nanofibrous scaffold based on gelatin/polyvinyl alcohol/chondroitin sulfate for cartilage regeneration by enhancing mesenchymal stem cell chondrogenesis differentiation on fabricated nanofibrous scaffold. After carrying out a cell viability assay, researchers discovered that the mesenchymal stem cells adhered and survived better on the nanofibrous scaffold and that the chondrogenic markers collagen type II and chondrogenic proteoglycan also performed better. The fabricated nanofibrous scaffold appears to be a promising material for cartilage tissue engineering, according to this research [80]. Shojarazavi et al. [81] fabricated an electrospun nanofibrous silk fibroin combined with alginate/cartilage extracellular matrix hydrogel for cartilage tissue regeneration. The results showed that increasing the alginate concentration enhanced the compression elastic properties, as well as water retention potential, degradability, cell viability, and aggrecan and collagen type II synthesis for the best hydrogel, promoting it as a nanocomposite scaffold for cartilage injury regeneration [81]. Chen et al. [82] designed a novel 3D porous electrospun polylactic acid combined with gelatin/chondroitin sulfate scaffold for cartilage tissue regeneration (Figure 3). *In vivo*, rabbit cartilage defects were created and the chondrogenic potential for fabricated nanocomposite scaffold was enhanced, and the chondrogenic markers collagen type II and chondrogenic proteoglycan were expressively improved. Even so, notable reductions in two essential inflammatory factors in fabricated nanocomposite scaffold confirmed inflammatory inhibitory activity, indicating the favored property of fabricated nanocomposite scaffold for cartilage tissue engineering and its immunoregulation ability [82].

### 5.3. Electrospun Nanofibrous Scaffolds for Cardiovascular Tissue Engineering

Cardiovascular diseases or cardiovascular-related diseases have very high rates and are steadily increasing [83]. Therefore, an immense amount of focus and industries are collaborating to find the most suitable scaffold to grow the vessels using tissue engineering. Researchers have made numerous suggestions for finding biomaterials for the scaffold and ensuring that they are biodegradable and biocompatible; however, in the case of cardiovascular tissue engineering, the function of the vessels, arteries, and veins must be taken into consideration, as well as the properties and characteristics of the vessels, which provide the platform for constructing the most appropriate scaffold [84–87]. The properties that are to be highly considered are the elasticity of the scaffold with the ability to withstand high pressures, especially for the arteries and veins closer to the heart, i.e., the coronary arteries and veins [84, 85]. There are several types of materials to make the scaffold since the vessels are made up of three layers each having different properties that allow the vessels to execute their functions. The three layers of the vessels to be considered when constructing the scaffold with the most suitable biomaterials are the tunica intima that contains connective tissue to provide flexibility [85–87]; the tunica media, which also happens to be the thickest layer that provides support for the vessel and is responsible for changes in blood pressure; and the tunica externa, which provides structural support and keeps the vessel from expanding to critical levels due to blood pressure [88]. All these factors and functions of the vessels mentioned should be taken into consideration when finding the most suitable scaffold that would house those layers and allow being fully grown to be delivered to the patient [87]. The materials that were suggested by researchers and scientists all provide promising results to fully grow the cardiovascular tissue and have higher rates of biodegradability today. Examples of the suggested polymers are collagen, polyamide, polyhydroxybutyrate, and silk [89, 90]. All of the listed polymers have characteristics of biocompatibility and high rates of biodegradability; furthermore, these polymers ensure the full growth of the layers and sustain their natural function. Another material had to be considered due to its properties that would provide a great scaffold construction and maintain the property and characteristics of the layers [91, 92].

Shin and colleagues used poly (lactic-co-glycolic acids) that are biodegradable and add them to electrospun mesh containing neonatal rat cellosaurus cell which resulted in growing five even layers of cells without any complications [93]. Tondnevis et al. [94] introduced that gelatin and single-walled carbon nanotubes were used with physicochemically and biologically modulated polyurethane nanofibers for myocardial infarction regeneration. Composite scaffolds with biomimetic physical behavior, such as blood vessels, have been created and their Young's modulus and ultimate strength managed to improve. Seven days of culture yielded a dense layer of myocardial myoblast and endothelial cells that was covered by a confluent and dense layer of nanofibrous surface, which is critical for cardiovascular tissue engineering. After the experiments were completed, it was determined that the fabricated scaffolds were suitable for cardiovascular tissue engineering applications [94]. Ahmadi et al. [95] fabricate structurally imitates the extracellular matrix of cardiac tissue using a variety of polyurethane—chitosan and carbon nanotube composite nanofibrous scaffolds with random and aligned orientation. Nanofibrous scaffolds were found to be biocompatible and viable when used with H9C2 cells. The results showed that the fabricated nanofibrous composite scaffolds were electroconductive and that aligned nanofibers could be considered promising nanoscale characteristics for the healing of infarcted myocardium in scaffolds with them [95]. Dimopoulos et al. [96] have produced tissue-engineered vascular scaffolds from polycaprolactone materials that replicate vessel's architecture and biomechanics. Mechanical properties of polycaprolactone scaffolds were especially in comparison to native vessels and commercial synthetic grafts. As a result, researchers discovered a three-layered tubular-shaped scaffold that was extremely hydrophobic. Moreover, an order of magnitude difference in elastic modulus was achieved, resulting in mechanical inhomogeneity. Finally, the polymeric scaffolds' toxicity evaluation revealed that the materials were safe and did not release any toxic and dangerous substances [96].

### 5.4. Electrospun Nanofibrous Scaffolds for Skin Tissue Engineering

Tissue engineering is sophisticated by itself, which can be easily implemented into medicine. However, skin tissue engineering is a sophistication of its own: researchers and scientists have struggled in finding the most suitable scaffold that will biodegrade as the healing process is completed [97, 98]. The complicated factor comes from the function of the skin itself, the first line of defense by keeping pathogens away from the internal tissues and organs, and other essential functions that the skin tissue provides [99]. The pursuit of finding the most suitable scaffold is not the only struggle and worry: researchers have kept in mind factors that have to do with the delivery of engineered tissue itself, such as infection while healing and scar formation. Although these factors have to be eliminated with skin tissue engineering, the correct form of the scaffold is rather important to maintain a successful delivery [100, 101]. The main approach of skin tissue engineering to overcome the struggle of finding the most suitable scaffold is to illuminate the disadvantages of autografting and allografting. Although these methods have had many successes in treating many patients with skin diseases, there is still a significant amount of disadvantages with those treatment methods. Even if researchers are trying to improve autografting and allografting, the focus is now shifted to the more promising skin tissue engineering that will eliminate the disadvantages and complications [102–104]. Researchers and scientists are mainly concerned about the rate of biodegradability with the mechanical properties to be as close as possible to the natural skin tissue; moreover, factors concerning the scaffolds of the skin tissue such as moisture maintenance, angiogenesis, and gas exchange are to be highly considered in the skin tissue engineering process [100, 104]. Liu et al. [105] presented a novel elastic submicron fiber scaffold electrospun from poly (e-caprolactone-co-lactide) (PLCL) and Pluronic for skin tissue engineering. Pluronic and PLCL were electrospun together. On all PLCL/Pluronic blended scaffolds, adipose-derived stem cells demonstrated superior cell adherence and proliferation capability when compared to PLCL. The adipose-derived stem cells on the blended scaffolds were extremely elongated and well merged with the surrounding fibers, confirming the PLCL/Pluronic scaffolds' good cytocompatibility. As a result, these mixed scaffolds have a promising future in the field of skin tissue engineering [105].

Agarwal et al. [67] produced an electrospun poly (glycidyl methacrylate) (ES-PGMA) scaffold with PXS64, a small-molecule antiscarring agent. PXS64, a lipophilic neutral counterpart of mannose-6-phosphate, has been demonstrated to block transforming growth factor b1 activation (TGFb1). TGFb1 is a growth factor, the main protein cytokine that regulates the expression of collagen I during wound healing and thereby governs the formation of collagen scarring tissue. The nanofibers were evaluated for their biocompatibility as a tissue engineering scaffold; also, their ability to activate TGFb1 in human dermal skin fibroblasts is inhibited [106].

Using the electrospinning approach, Liu et al. [107] created ethylene vinyl alcohol (EVOH) mats with metal or metal oxide nanoparticles (Ag, CuO, and ZnO). The results reveal that the best temperature for fabricating the materials is 40°C (±3°C). According to the antibacterial experiment results, 0.08 g/ml of metal/metallic oxide has the best antibacterial potential against Staphylococcus aureus. Furthermore, the three varieties of nanofiber mats' bacteriostatic loops have the biggest widths. Finally, cell multiplication on the three nanofiber mats follows a similar pattern [107].

Hadisi et al. [108] had successfully shown that by using *Lawsonia inermis* (also known as henna) in a scaffold composed of gelatin oxidized starch nanofibers, it aids with healing second-degree burns and decreases pathogen intrusion and inflammatory responses [108]. Movahedi et al. [109] fabricated a new polyurethane and hyaluronic acid nanofibrous scaffold for skin tissue engineering by coaxial electrospinning procedure. *In vitro* testing of nanofibers was done on mouse fibroblasts (L929), which showed that cellular morphology and viability improved significantly when the cells were promoted and attached. Additional research has shown that the nanofibrous mesh for wound dressing may be a suitable candidate for skin tissue engineering and wound healing [109]. Narayanan et al. [110] explored that the extracellular matrix can be mimicked for skin tissue engineering by using electrospun nanofibers of glucose-reduced graphene oxide that was reinforced with polyvinyl alcohol scaffolds and chemically crosslinked with acidic glutaraldehyde in an acetone medium. *In vitro* hemolytic, viability and proliferation assays with CCD-986Sk (a human skin fibroblast cell line) and live/dead cell imaging were used to evaluate the biological activities of nanofibrous scaffolds. In addition, the nanofibrous scaffold showed excellent compatibility with fibroblasts and significantly increased metabolic activity. The nanofibrous scaffolds increased fibroblast proliferation and viability in the presence of DAPI staining and live/dead imaging assays, leading to the possibility of skin tissue engineering [110]. Jiang et al. [111] fabricated sandwich scaffold that mimics the strain-strengthening activity of individual tissues. To begin, use wet electrospinning to create polycaprolactone yarns. After that, make a textile out of polycaprolactone yarns crocheted together (Figure 4). Finally, the sandwich scaffold is built by sandwiching the textile fabric between two electrospun mats. By using wet electrospun polycaprolactone yarns, you can induce cell alignment and lengthening in your research animals. The textile-based sandwich scaffold exhibits tensile-strengthening properties. After optimizing the thickness of the sandwich scaffold's outermost layer, the scaffold is also capable of supporting cell proliferation and infiltration. Textile-based sandwich scaffolds have the ability to mimic the physical, mechanical, and biological properties of human skin and other tissues, according to the findings of this study [111].

Widiyanti et al. [112] proposed a polycaprolactone with chitosan nanofibrous scaffold for skin tissue engineering. As a result, increasing the polycaprolactone concentration reduces the rate of degradation of the sample while increasing the sample contact angle (to measure sample surface wettability). It has been discovered that by studying the properties of chitosan-polycaprolactone composites, new products for skin tissue engineering can be developed that take advantage of these properties [112].

### 5.5. Electrospun Nanofibrous Scaffolds for Tendon and Ligament Tissue Engineering

The most common type of tendon injury is a rupture or tear, which can cause excruciating agony and necessitate up to 50 million surgical procedures per year [113, 114]. There is currently a viable approach for treating and regenerating injured tendons using tissue engineering scaffolds made of electrospun fibers [115].

Yang et al. [116] have produced an innovative, multiple-layered PCL/methacrylated gelatin composite scaffold with human adipose stem cell interspersions and double electrospinning. A methacrylated gelatin layer encased in five sheets of crosslinked polyethylene reinforced the scaffold. For 7 days, the human adipose stem cells were added with TGF-3 to encourage differentiation into tenocytes, and protein production assay revealed a significant increase in the expression of the tendon markers scleraxis and tenascin-C. A histone deacetylase inhibitor, trichostatin A, was electrospun into a scaffold by Zhang et al. [117] and tested for its effect on tenocyte development. The effects of trichostatin were greater in comparison to those of controls that did not use either the signaling molecule or random nanoplatforms. This study results showed significantly increased in tendon biomarkers expression and this study suggests that using trichostatin and topographical cues from aligned fibers could help promote tenolineage differentiation and repair of tendon defects. In order to create a tendon-to-bone interface, researchers used an electrospun mesh. Perikamana et al. [118] immobilized PDGF-BB on its aligned fibers in curves on its platelet-derived growth factor encourage adipogenic stem cell tenogenic development. PDGF-BB gradients on aligned nanofibers worked in concert with topographical signals to spatially govern cell differentiation, resulting in an anisotropic structure similar to the tendon-bone insertion site with lengthy cytoskeletons. These findings support the hypothesis. A 14-day study revealed that the scaffold enhanced the levels of biomarkers of tendon formation. According to these findings, a PDGF-BB gradient on aligned nanofibers could be effective for engineering the bone-tendon junction. Bone-tendon engineering may be improved by using aligned nanofibers coated with a PDGF-BB gradient. PLLA and PLLA layers filled with nanohydroxyapatite were used by Li et al. [119] to create a double-layer scaffold that mimicked enthesis fibrocartilage mineralized and nonmineralized. In *vivo* research, the double-layer scaffold demonstrated dramatically improvement in collagen production and increase in glycosaminoglycan exeprission at the tendon-bone interface site. Based on study findings, the bilayered scaffold may be useful for tissue engineering because it allows for precise control over the location of repair at the tendon-bone interface, mineralization and nonmineralization.

Sensini et al. [120] indicated that poly (L-lactic acid) and collagen electrospun scaffolds effectively promote different morphological changes in human fibroblasts in both static and dynamic cultures. The results showed that fibroblasts expanded on the external nanofibrous layer of the static scaffolds, elongating themselves circularly after 7 days of parallel cultures. The dynamic cultures demonstrated that fibroblasts develop preferentially axially on the exterior membrane. However, the aligned nanofiber bundles within the hierarchical scaffolds permitted for a natural distribution of fibroblasts along the nanofiber orientation. In another study, Sensini et al. [121] constructed morphological biomimetic hierarchical Nylon 6,6 electrospun bundles that mimic the function and structure of tendons and ligaments. The nanofibers in the solitary bundles and hierarchical arrangements exhibited shape and directionality identical to tendons and ligaments. The findings demonstrated an effective electrospinning production approach for constructing nanofibrous Nylon 6,6 hierarchical assemblies appropriate for future implanted devices and capable of mimicking the multiscale shape and biomechanical properties of tendons and ligaments.

## 6. Electrospun Nanofibers' Clinical Applications

Despite the fact that electrospinning is a simple, low-cost, and adaptable technology for generating fibrous scaffolds on a nanometer scale with huge promise for creating multifunctional materials used in tissue engineering, its therapeutic use has not yet been primarily managed in the market. Various companies have developed substantial technological advances in this field, but none of the products have yet received FDA approval [122, 123]. Nicast, for example, created AVflo™, a vascular access graft made of polycarbonate-urethane and silicone with a multilayered electrospun design [124]. Zeus® developed Bioweb™, an electrospun PTFE graft with applications in scaffolding, stent encapsulation, and embedded nanostructures in the body [125]. St. Teresa Medical, Inc.® constructed SURGICLOT®, a hemostatic dressing in which electrospun fibers release proteins to induce blood clotting, although it is not yet commercially accessible [126]. Aside from difficulties concerning the safety and efficacy of electrospun fibers, there are also economic and technical challenges that must be overcome in order to achieve their therapeutic uses. Along with an economic standpoint, electrospinning not only has a low productivity yield, but it also necessitates highly skilled workers to manufacture and develop high-quality products. Lack of advanced and comprehensive process and product quality control is a key issue from a technological standpoint. For example, large-scale commercial product production using an electrospinning setup in a continuous process remains difficult. By overcoming the aforementioned problems, the immense potential of electrospun nanofibers in tissue engineering can be realized and converted into clinical outcomes [127].

To overcome the limits of conventional techniques of tissue regeneration regarding precise control of scaffold pore size, geometry, and interconnectivity, recent breakthroughs in tissue engineering have applied three-dimensional (3D) printing, to fabricate bioscaffolds [128]. Tissue engineering can benefit from this technology's capacity to consistently 3D print many cell types in structured organizational regions, which makes this technology useful in this field. 3D bioprinting can be used to create multilayered skin, bone, vascular grafts, heart valves, and cartilage [129].

Whereas bioprinting has several benefits over traditional tissue engineering approaches, there are still integration and usage issues. For example, 3D-bioprinted tissue scaffolds have yet to be seen in real clinical settings because of inadequate mechanical characteristics and a lack of long data to indicate adequate biofabricated stability. These difficulties are also related to the types of cells and biomaterials used, as well as the bioprinting technology used [130]. There are numerous constraints of bioinks and bioprinters that make selecting an ink that shows all of the desired properties of a specific application challenging [7, 48]. The bioprinting technology chosen must be compatible with both the tissue being printed and the bioink used [128]. Furthermore, considering the high costs of 3D printers, cellular materials, and even computer software, the cost efficiency of 3D bioprinting must be examined. Overall, the costs of maintaining and expanding bioprinting technology make it difficult to bring 3D printing capabilities to clinics [131]. Moreover, the size of 3D-printed tissues is still a problem. Bioprinted tissues are currently tiny and made up of only a few cell types, resulting in limited functioning and scalability [132]. Despite significant research efforts to improve the manufacturing resolution of various types of 3D bioprinters, some challenges remain in the production of high-resolution 3D biostructures [133].

## 7. Conclusion and Future Prospects

Electrospun nanofiber scaffolds have recently emerged as a new alternative for tissue autologous grafts, the gold standard for tissue regeneration. Electrospun nanofiber scaffolds, as a fundamental component of tissue engineering, have the potential to be used in a wide range of tissues, including tendon, vascular, neuron, bone, and cartilage. On the one hand, for tissue repair, electrospun nanofiber scaffolds feature similarities to natural tissue and advantages such as high surface-to-volume ratio, variable porosity, and scale and shape similarity to the fibrous structure of natural extracellular matrix. Electrospun nanofiber scaffolds, on the other hand, come in a variety of designs for tissue regeneration.

Employing innovative nanomaterials combined with more favorable engineering techniques casts optimism brightness on the research area of tissue regeneration. Among the most versatile and attractive tools for producing a variety of nanostructured fibers is electrospinning. It has been used in a range of methods for combining material properties with various morphological properties for tissue engineering. Electrospun nanofibrous structures are more identical to the ECM nanostructure than other conventional methods. Numerous studies have shown that these advanced nanofibrous scaffolds work. Even so, additional *in vitro* and *in vivo* studies are required to fully define heretofore manufactured micro- and nanoscale fibers. Rather than contemplating designed nanofibrous scaffolds for biomedical technologies in general, researchers should point to definite scaffold uses by fine-tuning system functions to replicate the defined target cells and tissues. To enhance the mechanical behavior of electrospun nanostructures is critical, and it is a significant challenge that tissue engineers are currently experiencing. As a result, scientists are looking into polymer-ceramic composite fibers and thermal treatments to improve fiber bonding and it may be necessary to create 3D scaffolds with layered materials.

Electrospinning has been shown to be a valuable method for constructing tissue engineering scaffolds since it is simple, affordable, adaptable, and capable of creating ECM-mimicking structures. However, for ultimate clinical application, cell infiltration impediment, potential toxicity of solvents or crosslinkers, and insufficient mechanical strength of typical electrospun scaffolds should be studied. Also, electrospun nanofibers have showed promise in tissue engineering applications, but many technical challenges remain to be solved. The great bulk of published research has been conducted *in vitro*. As a result, the content and structure of polymeric nanofiber scaffolds still need to be further optimized for *in vivo* applications. Creating 3D porous scaffolds containing cells and growth factors is essential for future research on cell infiltration and survivability. Furthermore, it is critical to move electrospun nanofibers from the laboratory to the commercial scale. Despite numerous hurdles, electrospinning looks to be a promising technology for the manufacture of functional nanofibers, allowing researchers from various disciplines to design and produce innovative substrates for tissue engineering with desirable goals.

Future research should look into multifunctional scaffolds that, in addition to physically promoting cell development, also help with tissue regeneration by delivering bioactive signals. In contrast to conventional drug delivery, a combination of tissue engineering with drug delivery technologies results in site-specific drug release, which improves drug efficiency, reduces adverse effects, and protects unstable pharmaceuticals.

## Figures and Tables

**Figure 1:** Schematic representation of the general setup of electrospinning.

**Figure 2:** SEM images display the morphology and fiber diameter of PCL/gelatin nanofiber fabricated with different ratios (5 : 4 and 5 : 5)—(a, b) PCL/gelatin and (c, d) PCL/gelatin, respectively. (e, f) The optimized ratio (5 : 5) of PCL/gelatin/bioactive metal complex nanofiber morphology and diameter.

**Figure 3:** 3D electrospun scaffold fabrication schematic diagram. Coaxial electrospinning nanofiber membranes were cut into pieces and dispersed. The nanofiber dispersions were poured into a cylindrical mold and frozen and then freeze-dried for 2 hours at 180°C. The scaffold was then disposed of by water for SS fabrication.

**Figure 4:** Images of (a) a single chain and (b) multichain needle felted with various hook sizes. (c) Schematic illustration of manufacturing the sandwich scaffold's outermost layer by electrospinning on both sides of the woven material for the same period of time.

**Table 1:** Effects of electrospinning parameters on the morphology of electrospun fibers.

Parameter	Effect of parameter on fiber morphology
Viscosity/concentration	Fiber diameters increased with increasing concentration/viscosity.
Applied voltage	The relationship between voltage and fiber diameter was difficult to ascertain.
Distance between nozzle and collector	To acquire dry fibers, a minimum distance was needed. Also, beading was seen at either too close or too far distances.
Flow rate	Fibers with smaller diameters were produced at lower flow rates, and excessive flow rates resulted in fibers that were not dry when they arrived at the collector.
Solution conductivity	In general, higher conductivities resulted in smaller fibers, but increasing conductivity facilitated in the creation of bead-free fibers that were consistent.
Ambient parameters	As the temperature rose, the viscosity of the solution decreased, resulting in smaller fibers. Increasing humidity caused the fibers to develop circular pores.
Surface tension	As the surface tension coefficient of the solutions increased, the quantity of beads increased.

## Data Availability

The data used to support the findings of this study are included within the article.

## References

[1] Correia S. I., Pereira H., Silva-Correia J. (2014). Current concepts: tissue engineering and regenerative medicine applications in the ankle joint. *Journal of the Royal Society Interface*.

[2] Pina S., Ribeiro V. P., Marques C. F. (2019). Scaffolding strategies for tissue engineering and regenerative medicine applications. *Materials*.

[3] Saatchi A., Arani A. R., Moghanian A., Mozafari M. (2021). Synthesis and characterization of electrospun cerium-doped bioactive glass/chitosan/polyethylene oxide composite scaffolds for tissue engineering applications. *Ceramics International*.

[4] Lanza R., Langer R., Vacanti J. P., Atala A. (2020). *Principles of Tissue Engineering*.

[5] Berthiaume F., Maguire T. J., Yarmush M. L. (2011). Tissue engineering and regenerative medicine: history, progress, and challenges. *Annual Review of Chemical and Biomolecular Engineering*.

[6] Dzobo K., Thomford N. E., Senthebane D. A. (2018). Advances in regenerative medicine and tissue engineering: innovation and transformation of medicine. *Stem Cells International*.

[7] Geuens T., van Blitterswijk C. A., LaPointe V. L. (2020). Overcoming kidney organoid challenges for regenerative medicine. *NPJ Regenerative Medicine*.

[8] Fournier R. L. (2017). *Basic Transport Phenomena in Biomedical Engineering*.

[9] Ambekar R. S., Kandasubramanian B. (2019). Progress in the advancement of porous biopolymer scaffold: tissue engineering application. *Industrial & Engineering Chemistry Research*.

[10] Kumar R., Aadil K. R., Ranjan S., Kumar V. B. (2020). Advances in nanotechnology and nanomaterials based strategies for neural tissue engineering. *Journal of Drug Delivery Science and Technology*.

[11] Rahmati M., Mills D. K., Urbanska A. M. (2021). Electrospinning for tissue engineering applications. *Progress in Materials Science*.

[12] Bosworth L., Downes S. (2011). *Electrospinning for Tissue Regeneration*.

[13] Subbiah T., Bhat G. S., Tock R. W., Parameswaran S., Ramkumar S. S. (2005). Electrospinning of nanofibers. *Journal of Applied Polymer Science*.

[14] Angammana C. J., Jayaram S. H. (2016). Fundamentals of electrospinning and processing technologies. *Particulate Science and Technology*.

[15] Zhu W., Ma X., Gou M., Mei D., Zhang K., Chen S. (2016). 3D printing of functional biomaterials for tissue engineering. *Current Opinion in Biotechnology*.

[16] Lewis P. L., Shah R. N. (2016). 3D printing for liver tissue engineering: current approaches and future challenges. *Current Transplantation Reports*.

[17] Liu H., Ding X., Zhou G., Li P., Wei X., Fan Y. (2013). Electrospinning of nanofibers for tissue engineering applications. *Journal of Nanomaterials*.

[18] Sun B., Long Y. Z., Zhang H. D. (2014). Advances in three-dimensional nanofibrous macrostructures via electrospinning. *Progress in Polymer Science*.

[19] Okutan N., Terzi P., Altay F. (2014). Affecting parameters on electrospinning process and characterization of electrospun gelatin nanofibers. *Food Hydrocolloids*.

[20] Reneker D. H., Yarin A. L. (2008). Electrospinning jets and polymer nanofibers. *Polymer*.

[21] Li Z., Wang C. (2013). *Effects of working parameters on electrospinning*.

[22] Yang Q., Li Z., Hong Y. (2004). Influence of solvents on the formation of ultrathin uniform poly(vinyl pyrrolidone) nanofibers with electrospinning. *Journal of Polymer Science Part B: Polymer Physics*.

[23] Deitzel J. M., Kleinmeyer J., Harris D. E. A., Tan N. B. (2001). The effect of processing variables on the morphology of electrospun nanofibers and textiles. *Polymer*.

[24] Yang Y., Jia Z., Liu J. (2008). Effect of electric field distribution uniformity on electrospinning. *Journal of Applied Physics*.

[25] Yalcinkaya F., Yalcinkaya B., Jirsak O. (2016). *Dependent and independent parameters of needleless electrospinning. Electrospinning*.

[26] Rezaei A., Nasirpour A., Fathi M. (2015). Application of cellulosic nanofibers in food science using electrospinning and its potential risk. *Comprehensive Reviews in Food Science and Food Safety*.

[27] Haghi A. K., Akbari M. (2007). Trends in electrospinning of natural nanofibers. *Physica Status Solidi (a)*.

[28] Topuz F., Uyar T. (2020). Electrospinning of cyclodextrin nanofibers: the effect of process parameters. *Journal of Nanomaterials*.

[29] Rodoplu D., Mutlu M. (2012). Effects of electrospinning setup and process parameters on nanofiber morphology intended for the modification of quartz crystal microbalance surfaces. *Journal of Engineered Fibers and Fabrics*.

[30] Beachley V., Wen X. (2009). Effect of electrospinning parameters on the nanofiber diameter and length. *Materials Science and Engineering: C*.

[31] Greiner A., Wendorff J. H. (2007). Electrospinning: a fascinating method for the preparation of ultrathin fibers. *Angewandte Chemie International Edition*.

[32] Fridrikh S. V., Jian H. Y., Brenner M. P., Rutledge G. C. (2003). Controlling the fiber diameter during electrospinning. *Physical Review Letters*.

[33] Sukigara S., Gandhi M., Ayutsede J., Micklus M., Ko F. (2003). Regeneration of _Bombyx mori_ silk by electrospinning --part 1: processing parameters and geometric properties. *Polymer*.

[34] Yuan X., Zhang Y., Dong C., Sheng J. (2004). Morphology of ultrafine polysulfone fibers prepared by electrospinning. *Polymer International*.

[35] Casper C. L., Stephens J. S., Tassi N. G., Chase D. B., Rabolt J. F. (2004). Controlling surface morphology of electrospun polystyrene fibers: effect of humidity and molecular weight in the electrospinning process. *Macromolecules*.

[36] Pelipenko J., Kristl J., Janković B., Baumgartner S., Kocbek P. (2013). The impact of relative humidity during electrospinning on the morphology and mechanical properties of nanofibers. *International Journal of Pharmaceutics*.

[37] Liu Y., Liang W., Shou W., Su Y., Wang R. (2013). Effect of temperature on the crater-like electrospinning process. *Heat Transfer Research*.

[38] De Prá M. A. A., Ribeiro-do-Valle R. M., Maraschin M., Veleirinho B. (2017). Effect of collector design on the morphological properties of polycaprolactone electrospun fibers. *Materials Letters*.

[39] Park J. H., Braun P. V. (2010). Coaxial electrospinning of self-healing coatings. *Advanced Materials*.

[40] Tong H. W., Zhang X., Wang M. (2012). A new nanofiber fabrication technique based on coaxial electrospinning. *Materials Letters*.

[41] Na H., Chen P., Wong S. C., Hague S., Li Q. (2012). Fabrication of PVDF/PVA microtubules by coaxial electrospinning. *Polymer*.

[42] Ahmed F. E., Lalia B. S., Hashaikeh R. (2015). A review on electrospinning for membrane fabrication: challenges and applications. *Desalination*.

[43] Briggs T., Arinzeh T. L. (2014). Examining the formulation of emulsion electrospinning for improving the release of bioactive proteins from electrospun fibers. *Journal of Biomedical Materials Research Part A*.

[44] Xu X., Zhuang X., Chen X., Wang X., Yang L., Jing X. (2006). Preparation of core-sheath composite nanofibers by emulsion electrospinning. *Macromolecular Rapid Communications*.

[45] Wu J., Liu S., He L. (2012). Electrospun nanoyarn scaffold and its application in tissue engineering. *Materials Letters*.

[46] Ali U., Zhou Y., Wang X., Lin T. (2012). Direct electrospinning of highly twisted, continuous nanofiber yarns. *Journal of the Textile Institute*.

[47] Williams D. F. (2008). On the mechanisms of biocompatibility. *Biomaterials*.

[48] Khanna A., Zamani M., Huang N.F (2021). Extracellular Matrix-Based Biomaterials for Cardiovascular Tissue Engineering. *Journal of Cardiovascular Development and Disease*.

[49] Sharifianjazi F., Esmaeilkhanian A., Moradi M. (2021). Biocompatibility and mechanical properties of pigeon bone waste extracted natural nano-hydroxyapatite for bone tissue engineering. *Materials Science and Engineering: B*.

[50] Perez-Puyana V., Jiménez-Rosado M., Romero A., Guerrero A. (2020). Polymer-based scaffolds for soft-tissue engineering. *Polymers*.

[51] Sharma S., Sudhakara P., Singh J., Ilyas R. A., Asyraf M. R. M., Razman M. R. (2021). Critical review of biodegradable and bioactive polymer composites for bone tissue engineering and drug delivery applications. *Polymers*.

[52] Savina I. N., Zoughaib M., Yergeshov A. A. (2021). Design and assessment of biodegradable macroporous cryogels as advanced tissue engineering and drug carrying materials. *Gels*.

[53] Martins A., Chung S., Pedro A. J. (2009). Hierarchical starch-based fibrous scaffold for bone tissue engineering applications. *Journal of Tissue Engineering and Regenerative Medicine*.

[54] Qu H., Fu H., Han Z., Sun Y. (2019). Biomaterials for bone tissue engineering scaffolds: a review. *RSC Advances*.

[55] Haleem A., Javaid M., Khan R. H., Suman R. (2020). 3D printing applications in bone tissue engineering. *Journal of Clinical Orthopaedics and Trauma*.

[56] Amini A. R., Laurencin C. T., Nukavarapu S. P. (2012). Bone tissue engineering: recent advances and challenges. *Biomedical Engineering*.

[57] Burg K. J., Porter S., Kellam J. F. (2000). Biomaterial developments for bone tissue engineering. *Biomaterials*.

[58] Black C. R., Goriainov V., Gibbs D., Kanczler J., Tare R. S., Oreffo R. O. (2015). Bone tissue engineering. *Current Molecular Biology Reports*.

[59] Rao S. H., Harini B., Shadamarshan R. P. K., Balagangadharan K., Selvamurugan N. (2018). Natural and synthetic polymers/bioceramics/bioactive compounds-mediated cell signalling in bone tissue engineering. *International Journal of Biological Macromolecules*.

[60] Chocholata P., Kulda V., Babuska V. (2019). Fabrication of scaffolds for bone-tissue regeneration. *Materials*.

[61] Ansari M. (2019). Bone tissue regeneration: biology, strategies and interface studies. *Progress in Biomaterials*.

[62] Rajzer I., Rom M., Menaszek E., Pasierb P. (2015). Conductive PANI patterns on electrospun PCL/gelatin scaffolds modified with bioactive particles for bone tissue engineering. *Materials Letters*.

[63] Li C., Vepari C., Jin H. J., Kim H. J., Kaplan D. L. (2006). Electrospun silk-BMP-2 scaffolds for bone tissue engineering. *Biomaterials*.

[64] Samadian H., Mobasheri H., Azami M., Faridi-Majidi R. (2020). Osteoconductive and electroactive carbon nanofibers/hydroxyapatite nanocomposite tailored for bone tissue engineering: in vitro and in vivo studies. *Scientific Reports*.

[65] Preeth D. R., Saravanan S., Shairam M. (2021). Bioactive zinc(II) complex incorporated PCL/gelatin electrospun nanofiber enhanced bone tissue regeneration. *European Journal of Pharmaceutical Sciences*.

[66] Meka S. R. K., Jain S., Chatterjee K. (2016). Strontium eluting nanofibers augment stem cell osteogenesis for bone tissue regeneration. *Colloids and Surfaces B: Biointerfaces*.

[67] Meka S. R. K., Kumar Verma S., Agarwal V., Chatterjee K. (2018). In situ silication of polymer nanofibers to engineer multi-biofunctional composites. *Chemistry Select*.

[68] Rajzer I., Kurowska A., Jabłoński A. (2018). Layered gelatin/PLLA scaffolds fabricated by electrospinning and 3D printing- for nasal cartilages and subchondral bone reconstruction. *Materials & Design*.

[69] Meka S. R. K., Agarwal V., Chatterjee K. (2019). _In situ_ preparation of multicomponent polymer composite nanofibrous scaffolds with enhanced osteogenic and angiogenic activities. *Materials Science and Engineering: C*.

[70] Gautam S., Sharma C., Purohit S. D. (2021). Gelatin-polycaprolactone-nanohydroxyapatite electrospun nanocomposite scaffold for bone tissue engineering. *Materials Science and Engineering: C*.

[71] Caplan A. I., Elyaderani M., Mochizuki Y., Wakitani S., Goldberg V. M. (1997). Overview Principles of cartilage repair and regeneration. *Clinical Orthopaedics and Related Research*.

[72] Tuan R. S., Chen A. F., Klatt B. A. (2013). Cartilage regeneration. *The Journal of the American Academy of Orthopaedic Surgeons*.

[73] Athanasiou K. A., Darling E. M., Hu J. C. (2009). Articular cartilage tissue engineering. *Synthesis Lectures on Tissue Engineering*.

[74] Semitela Â., Girão A. F., Fernandes C. (2020). Electrospinning of bioactive polycaprolactone-gelatin nanofibres with increased pore size for cartilage tissue engineering applications. *Journal of Biomaterials Applications*.

[75] Chung C., Burdick J. A. (2008). Engineering cartilage tissue. *Advanced Drug Delivery Reviews*.

[76] Irawan V., Sung T. C., Higuchi A., Ikoma T. (2018). Collagen scaffolds in cartilage tissue engineering and relevant approaches for future development. *Tissue engineering and regenerative medicine*.

[77] Wise J. K., Yarin A. L., Megaridis C. M., Cho M. (2009). Chondrogenic differentiation of human mesenchymal stem cells on oriented nanofibrous scaffolds: engineering the superficial zone of articular cartilage. *Tissue Engineering Part A*.

[78] Li W. J., Tuli R., Okafor C. (2005). A three-dimensional nanofibrous scaffold for cartilage tissue engineering using human mesenchymal stem cells. *Biomaterials*.

[79] Sharifi F., Irani S., Azadegan G., Pezeshki-Modaress M., Zandi M., Saeed M. (2020). Co-electrospun gelatin-chondroitin sulfate/polycaprolactone nanofibrous scaffolds for cartilage tissue engineering. *Bioactive Carbohydrates and Dietary Fibre*.

[80] Irani S., Honarpardaz A., Choubini N., Pezeshki-Modaress M., Zandi M. (2020). Chondro-inductive nanofibrous scaffold based gelatin/polyvinyl alcohol/chondroitin sulfate for cartilage tissue engineering. *Polymers for Advanced Technologies*.

[81] Shojarazavi N., Mashayekhan S., Pazooki H., Mohsenifard S., Baniasadi H. (2021). Alginate/cartilage extracellular matrix-based injectable interpenetrating polymer network hydrogel for cartilage tissue engineering. *Journal of Biomaterials Applications*.

[82] Chen S., Chen W., Chen Y., Mo X., Fan C. (2021). Chondroitin sulfate modified 3D porous electrospun nanofiber scaffolds promote cartilage regeneration. *Materials Science and Engineering: C*.

[83] Moriyama I. M., Krueger D. E., Stamler J. (1971). *Cardiovascular diseases in the United States*.

[84] Vara D. S., Salacinski H. J., Kannan R. Y., Bordenave L., Hamilton G., Seifalian A. M. (2005). Ingenierie tissulaire applique aux vaisseaux sanguins : etat de l'art. *Pathologie Biologie*.

[85] Sell S. A., McClure M. J., Garg K., Wolfe P. S., Bowlin G. L. (2009). Electrospinning of collagen/biopolymers for regenerative medicine and cardiovascular tissue engineering. *Advanced Drug Delivery Reviews*.

[86] Bouten C. V. C., Dankers P. Y. W., Driessen-Mol A., Pedron S., Brizard A. M. A., Baaijens F. P. T. (2011). Substrates for cardiovascular tissue engineering. *Advanced Drug Delivery Reviews*.

[87] Lee A. Y., Mahler N., Best C., Lee Y. U., Breuer C. K. (2014). Regenerative implants for cardiovascular tissue engineering. *Translational Research*.

[88] Oh B., Lee C. H. (2013). Nanofiber for cardiovascular tissue engineering. *Expert Opinion on Drug Delivery*.

[89] Heydarkhan-Hagvall S., Schenke-Layland K., Dhanasopon A. P. (2008). Three-dimensional electrospun ECM-based hybrid scaffolds for cardiovascular tissue engineering. *Biomaterials*.

[90] Generali M., Dijkman P. E., Hoerstrup S. P. (2014). Bioresorbable scaffolds for cardiovascular tissue engineering. *EMJ Interventional Cardiology*.

[91] Rhodes N. (2004). Biocompatibility testing of tissue engineered products. *Vox Sanguinis*.

[92] Majid Q. A., Fricker A. T., Gregory D. A. (2020). Natural biomaterials for cardiac tissue engineering: a highly biocompatible solution. *Frontiers in Cardiovascular Medicine*.

[93] Shin H. J., Lee C. H., Cho I. H. (2006). Electrospun PLGA nanofiber scaffolds for articular cartilage reconstruction: mechanical stability, degradation and cellular responses under mechanical stimulation in vitro. *Journal of Biomaterials Science, Polymer Edition*.

[94] Tondnevis F., Keshvari H., Mohandesi J. A. (2020). Fabrication, characterization, and in vitro evaluation of electrospun polyurethane-gelatin-carbon nanotube scaffolds for cardiovascular tissue engineering applications. *Journal of Biomedical Materials Research Part B: Applied Biomaterials*.

[95] Ahmadi P., Nazeri N., Derakhshan M. A., Ghanbari H. (2021). Preparation and characterization of polyurethane/chitosan/CNT nanofibrous scaffold for cardiac tissue engineering. *International Journal of Biological Macromolecules*.

[96] Dimopoulos A., Markatos D. N., Mitropoulou A., Panagiotopoulos I., Koletsis E., Mavrilas D. (2021). A novel polymeric fibrous microstructured biodegradable small-caliber tubular scaffold for cardiovascular tissue engineering. *Journal of Materials Science: Materials in Medicine*.

[97] Mansbridge J. (2008). Skin tissue engineering. *Journal of Biomaterials Science, Polymer Edition*.

[98] Priya S. G., Jungvid H., Kumar A. (2008). Skin tissue engineering for tissue repair and regeneration. *Tissue Engineering Part B: Reviews*.

[99] Singh D., Singh D., Han S. S. (2016). 3D printing of scaffold for cells delivery: advances in skin tissue engineering. *Polymers*.

[100] Mohamed A., Xing M. M. (2012). Nanomaterials and nanotechnology for skin tissue engineering. *International Journal of Burns and Trauma*.

[101] Mac Neil S. (2008). Biomaterials for tissue engineering of skin. *Materials Today*.

[102] Ullah S., Chen X. (2020). Fabrication, applications and challenges of natural biomaterials in tissue engineering. *Applied Materials Today*.

[103] Molina M. I. E., Malollari K. G., Komvopoulos K. (2021). Design challenges in polymeric scaffolds for tissue engineering. *Frontiers in Bioengineering and Biotechnology*.

[104] Weng T., Wu P., Zhang W. (2020). Regeneration of skin appendages and nerves: current status and further challenges. *Journal of Translational Medicine*.

[105] Liu N. H., Pan J. F., Miao Y. E., Liu T. X., Xu F., Sun H. (2014). Electrospinning of poly (*ε*-caprolactone-co-lactide)/Pluronic blended scaffolds for skin tissue engineering. *Journal of Materials Science*.

[106] Agarwal V., Wood F. M., Fear M., Iyer K. S. (2017). Polymeric nanofibre scaffold for the delivery of a transforming growth factor *β*1 inhibitor. *Australian Journal of Chemistry*.

[107] Liu D., Zhang C., Dong G. (2019). Temperature-controlled electrospinning of EVOH nanofibre mats encapsulated with Ag, CuO, and ZnO particles for skin wound dressing. *Materials Research Express*.

[108] Hadisi Z., Nourmohammadi J., Nassiri S. M. (2018). The antibacterial and anti-inflammatory investigation of *Lawsonia Inermis* -gelatin-starch nano-fibrous dressing in burn wound. *International Journal of Biological Macromolecules*.

[109] Movahedi M., Asefnejad A., Rafienia M., Khorasani M. T. (2020). Potential of novel electrospun core-shell structured polyurethane/starch (hyaluronic acid) nanofibers for skin tissue engineering: _in vitro and in vivo evaluation_. *International Journal of Biological Macromolecules*.

[110] Narayanan K. B., Park G. T., Han S. S. (2020). Electrospun poly(vinyl alcohol)/reduced graphene oxide nanofibrous scaffolds for skin tissue engineering. *Colloids and Surfaces B: Biointerfaces*.

[111] Jiang C., Wang K., Liu Y., Zhang C., Wang B. (2021). Textile-based sandwich scaffold using wet electrospun yarns for skin tissue engineering. *Journal of the Mechanical Behavior of Biomedical Materials*.

[112] Widiyanti P., Gayatri D. B., Rudyardjo D. I. (2021). Synthesis and characterization scaffold chitosan/poly (*ε*-caprolactone) as candidate for skin tissue engineering in burns. *Malaysian Journal of Medicine and Health Sciences*.

[113] Bass E. (2012). Tendinopathy: why the difference between tendinitis and tendinosis matters. *International Journal of Therapeutic Massage & Bodywork*.

[114] Ljungqvist A., Schwellnus M. P., Bachl N. (2008). International Olympic committee consensus statement: molecular basis of connective tissue and muscle injuries in sport. *Clinics in Sports Medicine*.

[115] Hampson K., Forsyth N. R., El Haj A., Maffulli N. (2008). Tendon tissue engineering. *Topics in Tissue Engineering*.

[116] Yang G., Lin H., Rothrauff B. B., Yu S., Tuan R. S. (2016). Multilayered polycaprolactone/gelatin fiber-hydrogel composite for tendon tissue engineering. *Acta Biomaterialia*.

[117] Zhang C., Wang X., Zhang E. (2018). An epigenetic bioactive composite scaffold with well-aligned nanofibers for functional tendon tissue engineering. *Acta Biomaterialia*.

[118] Perikamana S. K. M., Lee J., Ahmad T. (2018). Harnessing biochemical and structural cues for tenogenic differentiation of adipose derived stem cells (ADSCs) and development of an _in vitro_ tissue interface mimicking tendon-bone insertion graft. *Biomaterials*.

[119] Li X., Cheng R., Sun Z. (2017). Flexible bipolar nanofibrous membranes for improving gradient microstructure in tendon-to-bone healing. *Acta Biomaterialia*.

[120] Sensini A., Cristofolini L., Zucchelli A. (2020). Hierarchical electrospun tendon-ligament bioinspired scaffolds induce changes in fibroblasts morphology under static and dynamic conditions. *Journal of Microscopy*.

[121] Sensini A., Gotti C., Belcari J. (2019). Morphologically bioinspired hierarchical nylon 6,6 electrospun assembly recreating the structure and performance of tendons and ligaments. *Medical Engineering & Physics*.

[122] Persano L., Camposeo A., Tekmen C., Pisignano D. (2013). Industrial upscaling of electrospinning and applications of polymer nanofibers: a review. *Macromolecular Materials and Engineering*.

[123] Shahriar S. M., Mondal J., Hasan M. N., Revuri V., Lee D. Y., Lee Y. K. (2019). Electrospinning nanofibers for therapeutics delivery. *Nanomaterials*.

[124] Ryan C. N., Fuller K. P., Larrañaga A. (2015). An academic, clinical and industrial update on electrospun, additive manufactured and imprinted medical devices. *Expert Review of Medical Devices*.

[125] Agarwal S., Wendorff J. H., Greiner A. (2008). Use of electrospinning technique for biomedical applications. *Polymer*.

[126] Nemati S., Kim S. J., Shin Y. M., Shin H. (2019). Current progress in application of polymeric nanofibers to tissue engineering. *Nano Convergence*.

[127] Stoddard R. J., Steger A. L., Blakney A. K., Woodrow K. A. (2016). In pursuit of functional electrospun materials for clinical applications in humans. *Therapeutic Delivery*.

[128] Matai I., Kaur G., Seyedsalehi A., McClinton A., Laurencin C. T. (2020). Progress in 3D bioprinting technology for tissue/organ regenerative engineering. *Biomaterials*.

[129] Cui X., Boland T., DD'Lima D., Lotz M. K. (2012). Thermal inkjet printing in tissue engineering and regenerative medicine. *Recent Patents on Drug Delivery & Formulation*.

[130] Tan B., Gan S., Wang X., Liu W., Li X. (2021). Applications of 3D bioprinting in tissue engineering: advantages, deficiencies, improvements, and future perspectives. *Journal of Materials Chemistry B.*.

[131] Zhang X., Zhang Y. (2015). Tissue engineering applications of three-dimensional bioprinting. *Cell Biochemistry and Biophysics*.

[132] Feinberg A. W., Miller J. S. (2017). Progress in three-dimensional bioprinting. *MRS Bulletin*.

[133] Midha S., Dalela M., Sybil D., Patra P., Mohanty S. (2019). Advances in three-dimensional bioprinting of bone: progress and challenges. *Journal of Tissue Engineering and Regenerative Medicine*.

